# Correlation of Serum M-CSF, CER, and TIMP-1 Levels with Liver Fibrosis in Viral Hepatitis

**DOI:** 10.1155/2022/6736225

**Published:** 2022-09-30

**Authors:** Hairong Yao, Xuan Yang, Man Yan, Xueqin Fang, Yange Wang, Hong Qi, Li Sun

**Affiliations:** ^1^Department of Cardiology, Xi'an No.3 Hospital, The Affiliated Hospital of Northwest University, Xi'an, Shaanxi 710018, China; ^2^Department of Infection, Xi'an No.3 Hospital, The Affiliated Hospital of Northwest University, Xi'an, Shaanxi 710018, China; ^3^Department of Hepatobiliary, Xi'an No.3 Hospital, The Affiliated Hospital of Northwest University, Xi'an, Shaanxi 710018, China

## Abstract

**Objective:**

This research is aimed at investigating the relationship between liver fibrosis in viral hepatitis and macrophage colony-stimulating factor (M-CSF), tissue inhibitor of matrix metalloproteinase (TIMP-1), and ceruloplasmin (CER) in serum level.

**Methods:**

Patients were randomly selected among those admitted to our hospital, and 60 healthy volunteers were chosen to serve as control participants. The levels of serum M-CSF, CER, and TIMP-1 were compared. According to the severity of their liver fibrosis, patients with CHB were separated into four groups: S1, S2, S3, and S4. Serum levels of M-CSF, CER, and TIMP-1 were correlated with liver fibrosis and hepatitis markers, and the diagnostic usefulness of the three indices was assessed with liver cirrhosis patients.

**Results:**

Increases in M-CSF and TIMP-1 in the CHB group but decreases in CER were statistically significant (*P* < 0.05). Serum levels of M-CSF, CER, TIMP-1, HA, PC-III, C-IV, and LN differed significantly across the four study groups (*P* < 0.05). Over time, as liver fibrosis worsened, we observed a progressive uptick in M-CSF, TIMP-1, LN, HA, C-IV, and PC-III levels and a progressive downtick in CER levels, with significant (*P* < 0.05) differences between the groups. There was a significant positive correlation between liver fibrosis and serum M-CSF, PC-III, TIMP-1, HA, LN, and C-IV levels in the CHB group (*P* < 0.05) and a significant negative correlation between serum CER and these same factors (*P* < 0.05). The AUC of 0.956 for diagnosing the S4 stage was greater than that of 0.857, 0.851, and 0.817 for M-CSF, CER, and TIMP-1, respectively.

**Conclusions:**

In CHB patients, the liver fibrosis degree is associated with the M-CSF, CER, and TIMP-1 levels, and the combined clinical detection of these three markers has better diagnostic significance.

## 1. Introduction

The liver is crucial to functioning several vital processes, including metabolism, immunity, coagulation, and many more. Long-term infection with the hepatitis B virus (HBV) is the primary cause of chronic hepatitis B (CHB) fibrosis, a multisystem chronic liver disease. However, HBV is not easy to clear, the patient's liver function inflammation is apparent, and it may progress to liver cirrhosis, which has become a significant public health problem. Proactive and efficient therapeutic approaches will slow the advancement of liver fibrosis to cirrhosis [1, 2]. Liver biopsy, an invasive procedure with limited clinical applicability, is still the gold standard for diagnosing liver fibrosis, and the biochemical and serological indicators are convenient and economical, which is a hotspot of current research [3].

Macrophage colony-stimulating factor (M-CSF) is composed of fibroblasts, activated macrophages, endometrial epithelial secretory cells, bone marrow stromal cells, vitamin D-activated osteoblasts, and activated vascular endothelial cells. Hepatic inflammatory responses are partly mediated by serum M-CSF, which has a role in the pathophysiology of hepatic fibrosis [4] by attracting and aggregating hepatic stellate cells. Ceruloplasmin (CER) is primarily metabolized in the liver. CER is a serum glycoprotein with 6 copper atoms per molecule, which is mainly synthesized in the liver. When liver function is damaged, especially liver failure, the level of CER in serum often decreases significantly. The primary function of CER is to combine with serum-free copper to complete the transport and metabolism process. Abnormal liver function will lead to abnormal serum CER levels, resulting in a series of cell and organ toxicity after copper deposition [5]. Excessive accumulation of extracellular matrix (ECM) in the liver is linked to liver fibrosis, and the ECM metabolism is related to matrix metal proteases (MMPs) and tissue inhibitors of metal proteases (TIMPs) [6]. Studies have shown that only TIMP-1 and TIMP-2 exist in the liver, while the specificity and sensitivity of TIMP-1 are superior to TIMP-2 in liver fibrosis diagnosis [7]. Studies have shown that TIMP-1 plays a role in the progression of liver fibrosis by degrading and transforming epithelial cells into mesenchymal cells [8]. Based on these findings, this research is aimed at offering a reference for clinical diagnosis of liver fibrosis progression by analyzing the blood levels of M-CSF, CER, and TIMP-1 in HBV-infected CHB patients. The report is as follows.

## 2. Materials and Methods

### 2.1. Research Subjects

From March 2017 to March 2020, a total of 115 CHB patients admitted to our hospital were selected. Following were the criteria for inclusion: (1) the pathological diagnosis of the liver biopsy was based on the Protocol for Prevention and Treatment of Viral Hepatitis [9], and the diagnostic criteria were following the Guidelines for Prevention and Treatment of Chronic Hepatitis B (2019 edition) [10]. (2) Hepatitis B surface antigen test was positive, and HBV infection history was longer than six months. (3) There were no contraindications to liver puncture. (5) Complete clinical data. Exclusion criteria are as follows: (1) abnormal liver function brought on by autoimmune liver disease, fatty liver, other viral hepatitis, and alcohol-related liver disease; (2) accompanied by malignant tumor; (3) patients with heart, kidney, and other serious diseases; (4) patients with blood system diseases; (5) patients with a previous history of liver surgery; (6) pregnant and lactation women; and (7) patients are taking anti-inflammatory, antifibrotic, immune-regulating drugs before enrollment. Liver fibrosis was divided into four stages: S1 was mild fibrosis, with 32 cases; S2 was moderate fibrosis, with 28 cases; S3 was advanced liver fibrosis, with 30 cases; and S4 was liver cirrhosis, with 25 cases. Sixty healthy volunteers were chosen as a control group for the same period. The Medical Ethics Review Board provided its approval for this investigation.

### 2.2. Observation Indicators

(1) General data collection is as follows: weight, height, gender, systolic blood pressure (SBP), diastolic blood pressure (DBP), and age of the CHB group and the healthy group were collected. The changes in SBP and DBP of the subjects were measured by a sphygmomanometer. Body Mass Index (BMI) = weight/height^2^ (international unit kg/m^2^). (2) After enrolling patients, 3 mL of fasting venous blood was obtained, and the upper serum was collected by centrifugation. This allowed us to measure the serum levels of M-CSF, CER, and TIMP-1. Enzyme-linked immunoadsorption (ELISA) was used to measure M-CSF and TIMP-1 in the serum. The kits were purchased from Rapid Bio Company, USA. The serum CER level was detected by the immunoturbidimetric method, and the instrument was an IMMAGE 800 automatic specific protein analysis system produced by Beckman Company in the United States, and supporting reagents were used. (3) Comparison of serum liver fibrosis indexes in the CHB group is as follows: After the patients were enrolled, 3 mL of fasting venous blood was taken, and the upper serum was collected by centrifugation. Enzymatic chemiluminescence immunoassay was used to detect type IV collagen (C-IV), laminin (LN) levels, hyaluronic acid (HA), and type III procollagen (PC-III); the kits were purchased from Roche Germany.

### 2.3. Statistical Analysis

For the statistical analysis, we utilized SPSS 20.0. *t*-test was employed on measurement data represented as *x* ± *s*. The rate (%) was calculated from the count data, and a *χ*^2^ test was performed. The association between serum levels of M-CSF, CER, and TIMP-1 and HA, PC-III, C-IV, and LN was analyzed using Pearson's correlation analysis. Serum M-CSF, CER, and TIMP-1 levels were analyzed in connection to liver fibrosis severity using Spearman's correlation. Using a ROC curve, we compared the diagnostic accuracy of serum M-CSF, CER, and TIMP-1 for the S4 stage; a difference at the *P* < 0.05 was considered significant.

## 3. Results

### 3.1. Comparison of General Data between CHB Group and Healthy Group

Table 1 shows no statistically significant differences between the CHB group and the healthy group concerning gender, age, body mass index, systolic blood pressure, or diastolic blood pressure (*P* > 0.05).

### 3.2. Comparison of Serum M-CSF, CER, and TIMP-1 Levels between CHB Group and Healthy Group

Table 2 shows that compared to the healthy controls, the CHB group had significantly higher serum M-CSF and TIMP-1 levels and significantly lower CER levels. These differences were statistically significant (*P* < 0.05).

### 3.3. Comparison of Serum M-CSF, CER, and TIMP-1 Levels in CHB Patients with Different Degrees of Liver Fibrosis

The levels of serum M-CSF, CER, and TIMP-1 varied significantly across the S1, S2, S3, and S4 groups (*P* < 0.05). As liver fibrosis progressed, the blood levels of M-CSF, TIMP-1, and CER changed over time, with statistically significant variations across all groups (*P* < 0.05), as indicated in Table 3.

### 3.4. Changes in Serological Markers of Liver Fibrosis in CHB Patients

Serum C-IV, LN, PC-III, and HA levels varied across the S1, S2, S3, and S4 groups in a statistically significant way (*P* < 0.05). The blood levels of HA, PC-III, C-IV, and LN steadily increased as liver fibrosis progressed, and statistically significant differences existed between all groups (*P* < 0.05), as shown in Table 4.

### 3.5. Correlation of Changes in Serum M-CSF, CER, and TIMP-1 Levels with Liver Fibrosis, HA, PC-III, C-IV, and LN

The serum M-CSF and TIMP-1 in the CHB group were positively connected with hepatitis A, B, C, and IV, liver fibrosis, and liver nodules severity (*P* < 0.05), respectively, as shown in Table 5 and Figures 1–4.

### 3.6. Analysis of the Diagnostic Value of Serum M-CSF, CER, and TIMP-1 Levels for the S4 Stage

ROC curve was used for analysis. The AUC of the three indicators combined to diagnose the S4 stage was 0.956, which was higher than the 0.857, 0.851, and 0.817 of using M-CSF, CER, and TIMP-1 for diagnosis alone, respectively, as shown in Figure 5 and Table 6.

## 4. Discussion

Liver cirrhosis is the outcome of liver fibrosis, a degenerative condition familiar to many types of viral hepatitis. A critical step in the development is the hepatic stellate cell (HSC) activation. Liver fibrosis develops when activated HSCs deposit their ECM-laden extracellular matrix into liver tissues, causing a shift in the matrix's constituent proteins [11]. Since liver fibrosis is reversible, early detection of the severity of the condition is crucial to developing an effective treatment strategy and improving the prognosis [12]. HA, PC-III, C-IV, and LN are essential indicators of liver fibrosis. Liver fibrosis is connected with the amount of extracellular matrix present, and HA is a critical component of the extracellular matrix [13]. LN is a noncollagenous structural glycoprotein deposited in a large amount in the space of hepatic sinusoidal endothelial cells during liver fibrosis; C-IV is the main component of the hepatic interstitial basement membrane and forms the basement membrane along the hepatic sinusoidal wall together with LN. The liver fibrosis degree is closely related to C-IV and LN [14]. PC-III is mainly degraded by type III procollagen and released into the blood, effectively reflecting collagen production levels [15]. In this study, significant differences were seen between the patients' S1, S2, S3, and S4 in terms of serum HA, PC-III, C-IV, and LN levels. Serum levels of HA, PC-III, C-IV, and LN increased as liver fibrosis progressed, showing that HA, PC-III, C-IV, and LN levels were connected to the degree of liver fibrosis in patients. Moreover, this finding has vital clinical guiding importance.

M-CSF is a cytokine produced by activated macrophages, endometrial epithelial secretory cells, osteoblasts, and other cells. By adhering to its receptors, it can control the proliferation and differentiation of mononuclear macrophage cells, which is crucial for physiological processes such as bone metabolism, mammary gland development, and ovarian ovulation; it can also be used as a proinflammatory cytokine to participate in inflammatory and immune responses and to participate in the pathological process of liver fibrosis [16, 17]. In this study, CHB had a greater serum M-CSF level than the healthy group. Between the S1, S2, S3, and S4 patient groups, there were considerable changes in the serum M-CSF levels, and the M-CSF rose dramatically as liver fibrosis progressed. The degree of liver fibrosis, HA, PC-III, C-IV, and LN levels were all positively linked with serum M-CSF levels, indicating a possible connection between the two. ROC curve analysis was used to determine the AUC of serum M-CSF for the diagnosis of the S4 stage, and it was determined to be 0.857, indicating that M-CSF can be used as a serological indicator for clinical diagnosis of liver cirrhosis. The reasons may be the following aspects: (1) M-CSF can regulate the expression of chemokines and receptors in monocytes and macrophages so that the inflammatory response of the liver continues. (2) The increased expression of M-CSF can regulate the production of MMP, aggravate the deposition of collagen fibers, and increase inflammatory cells infiltration in the liver. (3) M-CSF may prevent NK cells from producing and secreting antifibrotic factor (interferon), thereby reducing the apoptosis of HSC and indirectly promoting the progression of liver cirrhosis [18, 19].

CER is a single-chain *α*2 globulin with oxidase, mainly synthesized and secreted by the liver. When hepatocytes are immune-damaged by HBV replication in the body, the synthesis of CER will be reduced [20]. Studies have shown that [21] individuals with nonalcoholic fatty liver disease who have the CER gene mutation also have more severe liver fibrosis. Hyperferritinemia and increased hepatic iron storage have been linked to CER gene mutations in these patients. In this study, CHB had a lower serum CER level than the healthy group. Between the patient groups S1, S2, S3, and S4, the serum CER levels varied significantly, and the CER decreased significantly with the aggravation of liver fibrosis degrees. The serum CER levels were negatively correlated with C-IV, PC-III, LN liver fibrosis degree, and HA levels. According to ROC analysis, serum CER may be utilized as a sensitive biomarker for the diagnosis of liver cirrhosis, with an AUC of 0.851 for the diagnosis of the S4 stage. Tan et al. [22] have shown that in patients with CHB, CER levels correlated with the liver fibrosis degree, which was of great value in diagnosing CHB cirrhosis. Kang et al. [23] showed that patients with HBV infection have a negative correlation between CER and liver fibrosis. Significant fibrosis, advanced fibrosis, and liver cirrhosis were all predicted by CER with AUCs of 0.774, 0.812, and 0.853, respectively, which were similar to the results of this study.

TIMP-1 was firstly isolated from the skeletal muscle of rabbits. The encoding gene is located in the P11 region of the X chromosome and is secreted by HSCs. The TIMP levels were proportional to the number of activated HSCs [24]. There was a correlation between TIMP-1 levels and liver fibrosis severity and cirrhosis in patients with CHB [25]. According to a study by Medeiros et al. [26], patients with chronic hepatitis C who were treated with direct-acting antiviral therapy had significantly lower levels of MMP-9/TIMP-1, suggesting that this complex may be a valuable biomarker for active fibrosis that can determine the extent of liver fibrosis in patients following viral clearance. Serum TIMP-1 levels in CHB were greater than those in the control group. Significant variations in blood TIMP-1 levels were seen between the S1, S2, S3, and S4 groups of individuals. In a positive correlation with liver fibrosis, HA, PC-III, C-IV, and LN severity, TIMP-1 seemed to be linked to fibrosis progression. The area under the curve (AUC) for TIMP-1 in the diagnosis of the S4 stage was 0.817, according to ROC curve analysis, while the AUC of the combination of the three indicators was 0.956, which were all higher than the single indicator, suggesting that the combined diagnostic value of M-CSF, CER, and TIMP-1 was higher than using a single indicator for prediction. It primarily results from the fact that TIMP-1 can bind to all MMPs, except for MMP-14 and MMP-19, which may block the action of MMP-1, slow down the breakdown of ECM, and encourage the development of liver fibrosis [27]. Researchers have found that [28] cucurbitaside protects liver tissue and slows the progression of liver fibrosis in a mouse model. This protective effect might be due to cucurbitaside's ability to inhibit lipid peroxidation and collagen synthesis by reducing the expression of Col-I, TIMP-1, TIMP -2 mRNA, and MMP-2 TGF-1 proteins. Of course, this research still has certain shortcomings. This research only includes a small number of patients, and their inclusion may have been predetermined. An active investigation on the levels of M-CSF, CER, and TIMP-1 in CHB patients does not exist simultaneously. The evolution of these markers after therapy is not looked into. Future research will combine many locations to increase the number of samples used, enhancing the depth and precision of this investigation.

In conclusion, liver fibrosis is associated with M-CSF, CER, and TIMP-1 levels in CHB patients. The diagnostic significance of the clinical combination detection of these three indications is higher, which aids in clinical prevention and treatment.

## Figures and Tables

**Figure 1:** Correlation of changes in serum M-CSF, CER, and TIMP-1 levels and liver fibrosis degree.

**Figure 2:** Correlation of serum M-CSF levels with HA, LN, C-IV, and PC-III levels.

**Figure 3:** Correlation of CER serum levels with C-IV, PC-III, HA, and LN levels.

**Figure 4:** Correlation of serum TIMP-1 levels with C-IV, PC-III, HA, and LN levels.

**Figure 5:** ROC curve analysis of serum M-CSF, CER, and TIMP-1 levels for the diagnosis of the S4 stage.

**Table 1:** Comparison of general data between the two groups.

Group	Number of cases	Gender (male/female, cases)	Age (years)	BMI (kg/m^2^)	SBP (mmHg)	DBP (mmHg)
CHB group	115	69/46	46.57 ± 7.85	25.43 ± 4.61	127.87 ± 7.49	78.42 ± 6.37
Healthy group	60	31/29	46.32 ± 7.49	24.89 ± 4.97	128.20 ± 8.71	77.80 ± 6.78
*t*/*χ*^2^		1.118	0.203	0.716	0.261	0.598
*P*		0.290	0.839	0.475	0.794	0.551

**Table 2:** Comparison of serum M-CSF, CER, and TIMP-1 levels between the CHB group and healthy group.

Group	Number of cases	M-CSF (pg/mL)	CER (g/L)	TIMP-1 (*μ*g/L)
CHB group	115	241.83 ± 64.80	0.24 ± 0.08	175.15 ± 37.79
Healthy group	60	140.01 ± 42.28	0.30 ± 0.05	127.01 ± 22.95
*t*		11.003	5.291	9.030
*P*		<0.001	<0.001	<0.001

**Table 3:** Comparison of serum M-CSF, CER, and TIMP-1 levels in CHB patients with different degrees of liver fibrosis.

Group	Number of cases	M-CSF (pg/mL)	CER (g/L)	TIMP-1 (*μ*g/L)
S1 group	32	181.12 ± 36.82	0.31 ± 0.11	143.68 ± 23.09
S2 group	28	227.26 ± 52.17①	0.25 ± 0.05①	162.02 ± 21.63①
S3 group	30	266.93 ± 43.08①②	0.22 ± 0.04①②	189.41 ± 23.40①②
S4 group	25	305.72 ± 50.14①②③	0.18 ± 0.02①②③	213.03 ± 39.57①②③
*F*		39.443	19.299	35.152
*P*		<0.001	<0.001	<0.001

Note: ^①^ indicated *P* < 0.05 when compared with the S1 group; ^②^ indicated *P* < 0.05 when compared with the S2 group, *P* < 0.05; ^③^ indicated *P* < 0.05 when compared with the S3 group.

**Table 4:** Changes in serological markers of liver fibrosis in CHB patients.

Group	Number of cases	HA (ng/mL)	PC-III (*μ*g/mL)	C-IV (*μ*g/mL)	LN (ng/mL)
S1 group	32	77.09 ± 18.27	102.71 ± 23.02	83.73 ± 16.20	94.62 ± 17.43
S2 group	28	172.58 ± 22.54①	121.56 ± 21.64①	111.47 ± 21.82①	135.09 ± 18.72①
S3 group	30	363.26 ± 30.62①②	202.48 ± 31.50①②	172.65 ± 25.41①②	154.66 ± 25.89①②
S4 group	25	562.97 ± 41.75①②③	252.79 ± 27.16①②③	207.22 ± 34.75①②③	225.55 ± 31.34①②③
*F*		1399.680	216.987	138.553	153.927
*P*		<0.001	<0.001	<0.001	<0.001

Note: ^①^ indicated *P* < 0.05 when compared with the S1 group; ^②^ indicated *P* < 0.05 when compared with the S2 group, *P* < 0.05; ^③^ when compared to the S3 group, *P* < 0.05.

**Table 5:** Correlation of changes in serum M-CSF, CER, and TIMP-1 levels with the degree of liver fibrosis, HA, PC-III, C-IV, and LN.

Correlative factors	The degree of liver fibrosis		HA (ng/mL)		PC-III (*μ*g/mL)		C-IV (*μ*g/mL)		LN (ng/mL)	
	*r*	*P*	*r*	*P*	*r*	*P*	*r*	*P*	*r*	*P*
M-CSF	0.727	<0.001	0.691	<0.001	0.626	<0.001	0.651	<0.001	0.606	<0.001
CER	-0.606	<0.001	-0.515	<0.001	-0.482	<0.001	-0.525	<0.001	-0.479	<0.001
TIMP-1	0.685	<0.001	0.679	<0.001	0.652	<0.001	0.551	<0.001	0.628	<0.001

**Table 6:** A diagnostic value analysis of serum M-CSF, CER, and TIMP-1 levels for the S4 stage.

	AUC	*P* value	Cutoff value	Sensitivity	Specificity	95% CI
M-CSF	0.857^#^	<0.001	272.71 pg/mL	84.00	84.44	0.777~0.937
CER	0.851^#^	<0.001	0.21 g/L	96.00	75.56	0.782~0.919
TIMP-1	0.817^#^	<0.001	204.38 *μ*g/L	64.00	94.40	0.715~0.919
Combined	0.956	<0.001	—	96.00	83.33	0.922~0.991

Note: Compared with the prediction value by combined indicators, ^#^*P* < 0.05.

## Data Availability

The labeled dataset used to support the findings of this study are available from the corresponding author upon request.
